# *Citrus sinensis* and *Musa acuminata* Peel Waste Extract Mediated Synthesis of TiO_2_/rGO Nanocomposites for Photocatalytic Degradation of Methylene Blue under Visible Light Irradiation

**DOI:** 10.1155/2022/5978707

**Published:** 2022-01-25

**Authors:** Mulugeta Hirko Olana, Fedlu Kedir Sabir, Eneyew Tilahun Bekele, Bedasa Abdisa Gonfa

**Affiliations:** ^1^Applied Chemistry Department, College of Natural and Computational Science, Ambo University, P.O. Box 19, Ambo, Ethiopia; ^2^Department of Applied Chemistry, School of Applied Natural Science, Adama Science and Technology University, P.O. Box 1888, Adama, Ethiopia

## Abstract

Water pollution caused by various natural and artificial sources such as expansion of industrialization, rapid increment in population size, the threat of climate change, and development in urbanization takes a serious attention. Due to this fact, various protocols and techniques were adopted for the treatment of such polluted water. In the present findings, TiO_2_ nanoparticles (NPs) and TiO_2_/rGO nanocomposites (NCs) were synthesized using titanium tetra butoxide in the presence of *Citrus sinensis* (CS) and *Musa acuminata* (MA) peel waste extract as a capping, reducing, and stabilizing agent. The synthesized NPs and NCs were characterized using thermogravimetric-differential thermal analysis (TGA/DTA), X-ray diffraction (XRD), scanning electron microscope (SEM), high resolution transmission electron microscopy (HR-TEM), selected area electron diffraction (SAED) pattern, ultraviolet diffuse reflectance spectroscopy (UV-DRS), and Fourier transform infrared (FTIR) spectroscopy. The synthesized NPs and NCs were investigated as green alternative photocatalyst for the degradation of methylene blue (MB) dye under visible light irradiation. Thermal analysis results confirmed that the green synthesized TiO_2_ NPs were found to be too stable above 550°C. XRD analysis result showed that the average crystalline size of CS and MA mediated synthesized TiO_2_ NPs with various volume ratios was in the range of 7.3–27.3 nm and 13.4–22.4 nm, respectively. The average crystalline size of CS and MA peel extract template synthesized TiO_2_/rGO NCs was found to be in the range of 7.5–15.3 and 11.2–12.5 nm, respectively. The band gap energy was calculated to be in the range of 3.17–3.29 eV and 3.10–3.38 eV for the CS and MA mediated synthesized TiO_2_ NPs, respectively. *E*_*g*_ of CS and MA peel extract template formed TiO_2_/rGO NCs was found to be in the range of 2.85–3.11 eV and 3.07–3.11 eV, respectively. SEM analysis proved that the various synthesized TiO_2_ NPs and TiO_2_/rGO NCs were spherical in shape and the absence of any other foreign materials confirmed the purity of the corresponding nanocatalysts. In addition, TEM, HRTEM, and SAED analysis confirmed that the structures of the synthesized nanocatalysts were spherical in shape and the catalysts were too crystalline and the result was found to fit with the XRD result. Among the synthesized various volume ratios of TiO_2_ nanocatalysts, high percentage of degradation (62% and 58.2%) was achieved using TiO_2_-2c and TiO_2_-2 m, respectively. Moreover, 94.28% and 94.25% of MB degradation were achieved in the presence of TiO_2_/rGO-1.5c and TiO_2_/rGO-1.5c nanocomposite photocatalysts, respectively.

## 1. Introduction

The natural ecosystem has been exposed to various natural and artificial hazardous problems due to overpopulation growth, advancements in urbanization, accumulation of agricultural fruit and vegetable wastes and industrial wastes including organic dyes, pesticides, inorganic contaminants and detergents, and heavy and toxic metal ions, and the decomposition of toxic and poisonous gases and chemical species produced from various chemical industries. Among these, the discharge of various types and nature of dye effluents from various chemical industries and sources such as dye stuffs, textiles, paint and varnishes, inks, plastics, pulp and paper, food, rubber, and cosmetics to the environment is a prime cause of concern nowadays worldwide [1–3]. Thus, it has been reported that developing and designing of an efficient and convenient removal protocol of these various types of pollutants from wastewater is becoming an urgent and challenging issue worldwide [4, 5].

Currently, various semiconductor-based nanomaterials have attracted a significant interest for the purification and treatment of wastewater. Among these, nanosized metal oxide photocatalysts such as TiO_2_, CuO, Co_3_O_4_, ZnO, ZnS, CdS, Fe_2_O_3_, MgO, Mn_2_O_3_, ZrO_2_, V_2_O_5_, Nb_2_O_5_, and WO_3_ have been investigated and used in the process of wastewater decontamination. Particularly, wastewater decontamination using high surface area semiconductor nanocomposite photocatalysts prepared via numerous techniques has shown improved potential. Previously, it has been reported that TiO_2_ NPs has been abundantly used and selected as the most reliable candidate as an environmentally clean and pristine photocatalyst due to its desired chemical properties, favorable optical effects, chemically balanced and photochemical stability, dielectric properties, biological and chemical inertness, high redox potential, and good photocatalytic efficiency and nontoxicity [6–9]. Even though TiO_2_ NPs is a material of choice as effective photocatalyst candidate for the purification of water contains pollutants, several limitations such as fast recombination of photo excited electron-hole pairs, wide band gap energy (≈3.2 eV), and agglomeration have been reported [10]. This intern implies that single TiO_2_ nanocatalyst could tend to aggregate, agglomerate, narrow spectral band, and show high photo-generated charge recombination rate and this results in shrinking surface area and inferior photocatalytic performance and so lower degradation efficiency [11].

In order to improve and enhance the photocatalytic activity of TiO_2_ NPs, several approaches have been revised such as metallic and nonmetallic doping, conductive polymer doping, dye sensitization, and formation of composite by using various synthesis methods. Among these adapted techniques of preventing the electron-hole recombination rate, TiO_2_-based composite nanophotocatalysts are the most reliable and cost-effective candidates. Previously, TiO_2_-based nanocomposite materials such as TiO_2_/ZnO, g/TiO_2_, Bi_4_Ti_3_O_12_/Bi_2_Ti_2_O_7_, and Au/TiO_2_ were synthesized via various chemical synthetic protocols for photocatalytic applications [12, 13]. Various physicochemical synthesis protocols for TiO_2_-based nanocomposites including the green approach were also reported. Among these techniques, the green synthesis approach is ecofriendly, inexpensive, and easily manageable as it involves the use of green alternative starting materials (extract of plants, bacteria, algae, and fungi) as a template and green solvents such as ethanol and distilled water and nontoxic and less toxic precursors/salts [14].

*Citrus sinensis* represents the largest citrus cultivar groups grown around the world, accounting for 70% of the total annual production of *Citrus* species. *Citrus sinensis* peel waste is a rich source of various secondary metabolites which include flavonoids, steroids, hydroxyamides, alkanes, and fatty acids, coumarins, peptides, carbohydrates, carbamates, alkylamines, and carotenoids [15]. Similarly, *Musa acuminate* which is commonly called banana is herbaceous plant and belongs to the family of Musaceae. The plant is well known by its various bioactive compounds such as enzymes, polyphenol oxidase, pectin as gelling agent, vitamin A, gallocatechol, dopamine, vitamin E, vitamin B6, sitosterol, malic acid, succinic acid, and palmitic acid [16]. In addition to their medicinal usage for the treatment of various alignments and as sources of food, the peel part of the fruits could be accessed with zero cost and employed as a capping and reducing agent for the synthesis of various metal, metal oxides, composites, and doped nanomaterials for various applications.

Previously, several studies and reports have been focused on investigating the photocatalytic activity of chemically synthesized and to some extent green mediated obtained single TiO_2_ oxide NPs for the degradation of various organic pollutants for the remediation of polluted water caused by various sources. Moreover, earlier reports show that TiO_2_/rGO nanocomposites were synthesized by various chemical synthesis protocols for the remediation and recovery of wastewater contaminated by numerous sources. However, to the knowledge of us as researchers, still now there is not any scientific report on the green synthesis of TiO_2_/rGO nanocomposites in the presence of peel extract of *Citrus sinensis* and *Musa acuminata* as cost-effective capping and reducing agent for the efficient photocatalytic degradation of methylene blue dye. Furthermore, no previous comparative works were presented on the effect of *Citrus sinensis* and *Musa acuminata* peel waste extracts on the green alternative synthesis of TiO_2_/rGO NCs and their effect on the degradation of water pollutants. Therefore, the present work focuses and intensifies on the synthesis of TiO_2_ NPs and TiO_2_/rGO NCs within various volume ratios characterization and investigates the photocatalytic degradation of methylene blue dye under visible light irradiation.

## 2. Methodology

### 2.1. Chemicals and Reagents

The different chemicals, reagents, and solvents used during the present study include titanium tetra butoxide (Ti(OC_4_H_9_)_4_ 97%, Sigma-Aldrich), sulfuric acid (H_2_SO_4_ 98%, Sigma-Aldrich), phosphoric acid (H_3_PO_4_, 65%, Sigma-Aldrich), hydrochloric acid (HCl 36–38%, Sigma-Aldrich), hydrogen peroxide (H_2_O_2_ 30%, Sigma-Aldrich), potassium permanganate (KMnO_4_, Alpha), Barium chloride (BaCl_2,_ Alpha), methylene blue (C_16_H_18_ClN_3_S, LOBA Chemie), ethanol (C_2_H_5_OH 97%, Silva, Ethiopia), and graphite powder (diameter 6 mm, 99.995% trace metals basis, Sigma-Aldrich). All these chemicals were of analytical grades and were employed without any further purification.

### 2.2. Collection and Extraction of the Peel Wastes

The fresh and healthy fruits of *Citrus sinensis* (sweet orange) and *Musa acuminata* (banana) were collected from the local available market of Adama City, Oromia Region, Ethiopia. The collected samples were washed several times using distilled water to remove surface dust particles. Then, the peel parts were taken using knife and were allowed shadow drying. The peels were then grinded and packed in a glass bottle followed by covering with aluminum foil to avoid photooxidation. The extraction was carried out by taking 15 g of fine peel powder of each peel and then added into 500 mL conical flask separately followed by adding 250 mL of distilled water. Each of the mixtures of water and peel powder present in the separated conical flask was then boiled at a constant temperature of 70°C for 45 minutes and stirred using a magnetic stirrer at 1000 rpm and cooled to room temperature and filtered using watchman filter paper. Finally, the filtrates were stored at 4°C in a refrigerator for the synthesis of TiO_2_ NPs TiO_2_/rGO nanocomposites [17].

### 2.3. *Citrus sinensis* and *Musa acuminata* Peel Extract Mediated Synthesis of TiO_2_ NPs

TiO_2_ nanoparticles were synthesized via sol-gel method using titanium tetra butoxide as a precursor in the presence of *Citrus sinensis* and *Musa acuminata* as capping and reducing agent in three different volume ratios (1 : 2, 1 : 1, and 2 : 1). In typical reaction, 0.25 M of 40, 50, and 60 mL of C_16_H_36_O_4_ titanium precursor solutions were added into three different Erlenmeyer flasks followed by stirring for 30 minutes to maintain homogeneity. Then, in each Erlenmeyer flask containing the precursor solution, 60, 50, and 40 mL of *Citrus sinensis* peel extract were added drop by drop, respectively, and labeled as 1 : 2 (TiO_2_-0.5c), 1 : 1 (TiO_2_-1c), and 2 : 1 (TiO_2_-2c). The reaction mixtures were stirred for 5 hours using magnetic stirrer at room temperature. Then, afterward, 17 mL of 1 M NaOH solution was added dropwise to facilitate precipitation and was stirred for 30 minutes in order to maintain the homogeneity of the solution and the formed suspensions were kept at 4°C in a refrigerator overnight for further use. The three different volume ratio suspensions were then centrifuged three times at 4000 rpm followed by washing three times using distilled water and absolute ethanol followed by collecting using crucible ceramic dish and then oven dry. The thermal stability of the dried samples was tested by taking the 1 : 1 ratio from each of the peel waste mediated synthesized TiO_2_ samples. Based on the thermal stability result, the three ratios of *Citrus sinensis* peel extract mediated synthesized TiO_2_ NPs were calcined at 500°C for 4 hours [18]. The same protocol was followed for the *Musa acuminata* peel extract mediated synthesis of TiO_2_ NPs and labeled as 1 : 2 (TiO_2_-0.5 m), 1 : 1 (TiO_2_-1 m), and 2 : 1 (TiO_2_-2 m).  Figure 1 shows the schematic synthetic procedure of TiO_2_ NPs in the presence of *Citrus sinensis* peel waste extract.

### 2.4. Synthesis of Graphene Oxide (GO)

Synthesis of GO was carried out following the modified tour method [19]. The synthesis procedure involved oxidation of graphite using strong oxidizing agent (KMnO_4_) in the presence of H_3_PO_4_ to prevent further possible oxidation [20]. Then, afterwards, 0.5 g of graphite powder was exfoliated using 90 mL of H_2_SO_4_ followed by addition of 50 mL *Citrus sinensis* peel waste extract in the presence of H_3_PO_4_ at 0°C in ice bath followed by gradual and stepwise addition of 4.5 g KMnO_4_. Then, the components were stirred for 8 hours while heating at 50°C using a temperature-controlled water bath. As the reaction time was extended and increased, the mixture turned out to paste. The reaction was then terminated by the addition of 250 mL of distilled water followed by addition of 10 mL H_2_O_2_ (30%) solution to reduce residual KMnO_4_ to soluble manganese sulfate (MnSO_4_) in an acidic medium. The formed suspension was then filtered to remove the metal sulfate and a graphite oxide filter cake was produced. The cake was then again washed using 5% of HCl until the sulfate ions are completely removed, which was confirmed using BaCl_2_ solution. The formed graphite oxide was washed three times at each centrifugation process at 1000 rpm for 30 minutes. The collected graphite oxide was added to 100 mL of distilled water and stirred followed by heating at 60°C for 8 hours in water bath. The brown colored GO solution was dried at 60°C for 6 hours in oven drier.  Figure 2 displays the resulting schematic synthesis protocol of rGO in the presence of peel waste extract of *Citrus sinensis* as a green alternative template.

### 2.5. *Citrus sinensis* and *Musa acuminata* Peel Extract Mediated Synthesis of TiO_2_/rGO Nanocomposites

The TiO_2_/rGO nanocomposites were prepared using synthesized GO and TiO_2_ via precipitation method in the presence of peel waste extract of *Citrus sinensis* (CS) and *Musa acuminata* (MA) as both reducing and stabilizing agent [21]. In a typical procedure, GO suspension was prepared by dispersing dried 30, 60, and 90 mg powders in 100 mL of distilled water by the process of sonication. Subsequently, 60 mg of TiO_2_ and 50 mL of CS extract were added into the GO slurry and stirred for 8 h at room temperature. Then, the solution turned to gray from brown colors indicating the reduction of GO to reduced graphene oxide (rGO). The gray residue of the formed rGO/TiO_2_-0.5c, rGO/TiO_2_-1c, and rGO/TiO_2_-1.5c nanocomposites was then centrifuged for a minimum of 30 minutes followed by washing three times using distilled water and absolute ethanol sequentially at each step of centrifugation to remove impurities. The obtained nanocomposites were then kept in vacuumed oven at 100°C for 24 hours for further analysis. The same procedure was followed for the *Musa acuminata* peel extract mediated synthesis and labeled as TiO_2_/rGO-0.5 m, TiO_2_/rGO-1 m, and TiO_2_/rGO-1.5 m nanocomposites.

### 2.6. Characterization

The thermal stability analysis study was done using a simultaneous TGA-DAT (DTG-60H, SHIMADZU Corporation, Japan). The crystal structure, average crystalline size, and phase stability of synthesized TiO_2_ NPs and TiO_2_/rGO nanocomposites were analyzed by XRD (XRD-7000, SHIMADZU Corporation, Japan) equipped with a Cu target for generating a Cu K*α* radiation with *λ* = 0.15406 nm and recorded in the range from 10°C to 80°. The morphological structure of each type of synthesized NPs and NCs was investigated using SEM. For further analysis and insights, the synthesized TiO_2_ NPs and TiO_2_/rGO nanocomposites were characterized using TEM, HRTEM, and SAED techniques. The optical property of both TiO_2_ NPs and TiO_2_/rGO nanocomposites was studied using UV-DRS (OPTIMA UV-Vis spectrometer SP-3000 Plus, SHIMADZU Corporation, Japan). Functional group analysis was studied using FTIR (FT/IR-6600 type A, JASCO Company, Japan) characterization techniques. The photocatalytic degradation studies of TiO_2_ and TiO_2_/rGO nanocomposites were carried out in 125 ml of Pyrex flask type reactor under 150W halogen lamp irradiation. The degradation analysis was followed and recorded using double beam UV-visible spectrophotometer (SM-1600 spectrometer MAALAB, India).

## 3. Results and Discussion

### 3.1. TGA/DTA Analysis

Figures 3(a) and 3(b) show the TGA/DTA of TiO_2_ synthesized using peel extract of *Citrus sinensis* and *Musa acuminate* of a 1 : 1 volume ratio, respectively. As presented in Figures 3(a) and 3(b), weight losses were observed in three stages for the TiO_2_ NPs synthesized using both peel extracts.

The first stage weight loss observed between 40 and 194°C was attributed to the removal of physically and chemically entrapped water and other moisture contents from the surface of the synthesized TiO_2_ nanoparticles. The second stage weight loss observed in the range of 195–503°C could be attributed to the losses of organic residues and organic molecules/compounds as a result of combustion and carbonization of biomass materials from the synthesized TiO_2_ NPs. Furthermore, no considerable weight loss was observed above 510°C which proved that the synthesized TiO_2_ NPs using *Citrus sinensis* (Figure 3(a)) and *Musa acuminata* (Figure 3(b)) peel waste extract was found to be nearly pure and thermally stable and hence temperature of 550 °C was selected as a calcination temperature [22–24].

### 3.2. XRD Analysis

Figure 4 depicts the XRD patterns of TiO_2_ NPs and TiO_2_/rGO NCs synthesized using various volume ratios of *Citrus sinensis* and *Musa acuminata*. As observed from Figures 4(a) and 4(b), TiO_2_-0.5c, TiO_2_-1c, TiO_2_-1.5c, TiO_2_-0.5 m, TiO_2_-1m, and TiO_2_-1.5 m showed diffraction peaks at 2*θ*≈25.3°, 38.4°, 48.55°, 55.55°, 62.66°, 69.77°, and 75.29° indexed to the crystalline planes of (101), (004), (200), (105), (204), (116), and (215), respectively. This corresponds to the standard pattern of the anatase crystalline phase form of TiO_2_ NPs with JCPDS card number of 21-1272 with tetragonal structure. The absence of any foreign materials and secondary phases is an indication of the high purity and stability of the NPs and NCs synthesized using fruit peel waste extracts. The various volume ratios of TiO_2_ NPs, TiO_2_-0.5c, and TiO_2_-0.5 m NPs showed less crystalline nature as compared to the other volume ratios due to the large amount of the peel extracts used which is in good agreement with previous report [25]. The average crystalline size of the synthesized NPs from various volume ratios was calculated using Debye Scherrer equation [26] and was found to be 27.3, 12.1, and 7.3 nm for the TiO_2_-0.5c, TiO_2_-1c, and TiO_2_-2c and 22.4, 16.3, and 13.4 nm for TiO_2_-0.5 m, TiO_2_-1 m, and TiO_2_-2 m, respectively.

Figures 4(c) and 4(d) provide the XRD pattern of *Citrus sinensis* and *Musa acuminata* peel extract synthesis of TiO_2_-1c, TiO_2_/rGO-1c, GO, TiO_2_-1 m, GO, and TiO_2_/rGO-1 m, respectively. It was found that the synthesized TiO2-rGO NCs possess a diffraction pattern similar to that of a single TiO_2_ NPs. Due to the small quantity and low intensity of rGO, there was no separate peak for the rGO within the TiO_2_-rGO NCs [27]. Previously, similar results were reported for the TiO_2_-activated carbon nanocomposites [28]. In addition to this, in both of the peel waste extracted mediated syntheses, the low peak intensity was due to the incomplete oxidation of graphite oxide and the cluster of bioactive constituents of the peel waste extract of *Citrus sinensis* and *Musa acuminata* added during the synthesis process [27–30].

Figures 4(e) and 4(f) present *Citrus sinensis* and *Musa acuminata* mediated synthesized TiO_2_, TiO_2_-rGO, and GO. The resulting diffraction pattern of GO showed a broad and relatively strong characteristic peak at 2*θ*≈10.1°, corresponding to the (001) plane, and this indicates the formation of GO sheets. The calculated average crystalline size of GO was found to be 9.8 nm. The spacing between GO sheets was attributed to the presence of oxygen functional groups such as hydroxyl, carboxyl, and epoxide groups on the carbon backbones as supported by the previously reported work [29]. In both of the peel waste extract mediated synthesized GO sheets, an incomplete oxidation of graphite powder was exhibiting a strong and sharp diffraction peak at 26.1°, which in turn is corresponding to the (002) plane [30].

### 3.3. SEM Analysis

Figures 5(a) and 5(b) clearly depict that the obtained rGO shows a wrinkled and crumpled morphology which is stacked together and forms a typical multilayer structure. This multilayer structure of rGO is important in providing additional rough surface for the deposition of *Citrus sinensis* and *Musa acuminate* template synthesized TiO_2_ NPs into rGO [31].

Figures 5(c)–5(h) show the SEM images of TiO_2_-0.5c, TiO_2_-1c, TiO_2_-2c, TiO_2_-0.5 m, TiO_2_-1 m, and TiO_2_-2 m NPs, respectively, and the images were found to possess spherical shaped surface morphology in the presence of distinct edges having wide rough surface. In both of the peel waste extract mediated synthesized TiO_2_ NPs using different volume ratios, the particle size was found to be increased with an increase in the amount of the peel waste extracts, which is in agreement with the calculated average crystalline size from the XRD analysis. Furthermore, homogenized and small particle size TiO_2_ NPs was obtained while using peel extract of *Citrus sinensis* due to its richness in biomolecules [32–34].

Moreover, Figures 5(i)–5(n) show the corresponding SEM images of TiO_2_/rGO-0.5c, TiO_2_/rGO-1c, TiO_2_/rGO-1.5c, TiO_2_/rGO-0.5 m, TiO_2_/rGO-1 m, and TiO_2_/rGO-1.5 m NCs, respectively. As can be observed from Figures 5(a) and 5(b), the rGO shows the wrinkled and crumpled morphology, while the *Citrus sinensis* and *Musa acuminate* based synthesized nanocomposites showed cross-linked TiO_2_ nanoparticles on the surface of the rGO sheet that formed the network structures within the rGO/TiO_2_ nanocomposites. It has been found that as the amount of rGO content is small, images of reduced graphene oxide-modified TiO_2_ NCs do not show a clear-cut presence of rGO flakes; rather it shows the uniform distribution of TiO_2_ NPs. The uniform distribution of TiO_2_ NPs is due to very small amount of rGO with respect to TiO_2_ NPs and intercalation of rGO inside the TiO_2_ NPs matrix [33]. However, as the content of rGO is increased from 30 to 90 mg, the size becomes clearly visible and this provides more surfaces for the deposition of green synthesized TiO_2_ NPs, which in turn is necessary for the photocatalytic degradation of MB dye.

The differences in the photocatalytic performance of those various compositions of TiO_2_/rGO NCs obtained in the presence of peel waste extracts of *Citrus sinensis* and *Musa acuminata* could be attributed to the amount of rGO to TiO_2_ composition ratio, in addition to the differences in the morphological structure [34].

### 3.4. TEM-HRTEM and SAED Pattern Analysis

Figures 5(a)–5(d) show TEM micrographs of *Citrus sinensis* mediated obtained TiO_2_NPs (a) and TiO_2_/rGO (b) and *Musa acuminata* peel waste obtained TiO_2_ NPs (c) and TiO_2_/rGO NCs (d). The TEM images of these peels waste extracted mediated synthesized TiO_2_ NPs using various volume ratios reveal that the nanoparticles were found to have good crystalline nature without aggregations and agglomerations. This is in agreement with the XRD results and in turn confirms the formation of pure TiO_2_ NPs [35, 36]. The absence of aggregations and agglomerations was achieved due to the presence of bioactive capping and reducing agents from the peel waste extract of *Citrus sinensis* and *Musa acuminata*. Furthermore, it can be observed from Figures 5(c) and 5(d) that rGO is found to be covered with the green synthesized spherical anatase TiO_2_ nanoparticles. The presented figures also showed crumpled, hexagonal, and rhombic-like large surface morphological structure due to the presence of the high surface area of the rGO sheets. It is also observed that the surface of rGO sheets was found to be packed densely with the green obtained TiO_2_ NPs which showed good combination of rGO sheets and TiO_2_ NPs and efficient TiO_2_ NPs loading on the surface sheet of rGO [37, 38].

The corresponding HRTEM images in Figures 5(e)–5(h) clearly showed that the lattice fringes of the rGO were parallel to the edges of the anatase TiO_2_ nanoparticles. The lattice fringes also clearly indicate that the particles are nanocrystalline with an anatase phase form as it is also confirmed from the XRD data. The figures indicated that the reduced graphene particles were well doped in the presence of the peel waste extracts with a dense layer of TiO_2_ nanocomposites having d-spacing value of 0.3, 0.33, 0.35, and 0.31 nm for the TiO_2_/*Musa acuminata* (e), TiO_2_/*Citrus sinensis* (f), TiO_2_/rGO/*Musa acuminata* NCs (g), and TiO_2_/rGO/*Citrus sinensis* NCs, respectively, corresponding to the d_101_ of TiO_2_ anatase structured NPs. The slight variation in the d-spacing value of TiO_2_ NPs and TiO_2_/rGO NCs may result from the presence of various bioactive molecules of the *Musa acuminata* and *Citrus sinensis* [39].

Figures 6(i)–6(l) present SAED pattern of the green synthesized TiO_2_ NPs and TiO_2_/rGO NCs obtained in the presence of the peel waste extract of *Citrus sinensis* and *Musa acuminata*. Figures 6(i)–6(j) showed the SAED of TiO_2_ NPs obtained using *Citrus sinensis* and *Musa acuminata* peel extract and the resulting SAED pattern proves the presence of clear ring diffraction patterns and does not indicate the presence of any dislocations in the lattice planes, which confirms that the prepared TiO_2_ nanoparticles have high crystallinity nature. The clear white circular spots around the center of SAED pattern confirm (101), (004), (200), (105), (211), (204), (220), and (215) miller indices as also supported by the XRD analysis assuring anatase lattice planes of biosynthesized TiO_2_ nanoparticles. Similarly, Figures 6(k) and 6(l) indicate the SAED analysis of the TiO_2_/rGO/*Musa acuminata* and TiO_2_/rGO/*Citrus sinensis* NCs, respectively, and similar pattern was observed as in the case of the single green synthesized TiO_2_ NPs [40, 41].

### 3.5. UV-DRS Analysis

Figures 7(a)–7(f) show the UV-DRS absorption spectra of TiO_2_ NPs prepared using different volume ratios of titanium precursor salt and peel waste extract of *Citrus sinensis* (a-c) and *Musa acuminata* (d–f). The optical band gap energy for each of the volume ratios of TiO_2_ NPs was calculated using Tauc plot method. The band gap energy (*E*_*g*_) was found to be 3.17, 3.28, 3.29, 3.10, 3.33, and 3.38 eV for the TiO_2_-0.5c, TiO_2_-1c, TiO_2_-2c, TiO_2_-0.5 m, TiO_2_-1 m, and TiO_2_-2 m, respectively. This is again found to be in close agreement with the work reported by Bekele [25].

As presented in Figure 7, it was found that increasing rGO concentrations in the composite tends to decrease energy band gap in each of the peel waste extract mediated synthesized TiO_2_/rGOs. In addition to this, it is noted that the presence of rGO influences light absorption properties of the composite significantly showing increase in light absorption intensity in the UV region and a red shift in the absorption edge around 400 nm as supported by the previous report [42]. Furthermore, the TiO_2_/rGO nanocomposites show a red shift in the absorption edge compared to single TiO_2_ NPs. Similar phenomenon related to the present study was also reported by Zhang et al. [43].

### 3.6. FT-IR Analysis

As depicted in Figure 8(a), the peel extract of *Citrus sinensis* shows various absorption bands, stretching, and bending mode of vibration located at 3447.81, 2920.53, 2327.68, 1637.89, 1449.65, and 1076.51 cm^−1^ and similarly *Musa acuminata* peel waste powder shows various absorption peeks located at 3433.64, 2920.50, 2324.60, 1639.52, 1405.71, and 1090.65 cm^−1^. In both cases of the peel waste extract, the broad band at 3447.81 and 3433.64 cm^−1^ is assigned to hydrogen bonded-OH stretching mode of vibration. The bands centered at 2920.53 and 2920.50 cm^−1^ represent H-C-H, C-H bond stretching of alkanes and -C-H groups associated with H-bond [44]. The week band observed at 1639.52 and 1641.73 cm^−1^ is attributed to the amide group vibration, which could be a characteristic peak of both proteins and enzymes present in both of the peel extracts [45]. Figures 8(a) and 8(b) also show stretching vibrations located at 1405.71 and 1449.65 cm^1^ for the *Citrus sinensis* and *Musa acuminata* peel extract, respectively, which indicates the binding of proteins on the surface of TiO_2_ NPs and thereby contributes to the stabilization of green TiO_2_ NPs. The bands observed at 1090.65 and 1076.55 cm^−1^ for *Citrus sinensis* and *Musa acuminata*, respectively, indicate the presence of C-O and aliphatic amines [46].

Figures 8(a) and 8(b) also show the corresponding FTIR spectra of GO and rGO. GO displayed numerous typical absorption bands corresponding to oxygen functionalities present on GO sheet. The band at 1725 cm^−1^ is credited to the C=O and the wide band around 3000–3600 cm^−1^ is ascribed to the O-H (hydroxyl) stretching vibrations of the C-OH groups due to moisture absorbed onto the surface of prepared sample. The band corresponding to 1056 cm^−1^ and 1248 cm^−1^ are credited to C-O (carboxylates) and C-O-C (epoxide) stretching modes, respectively. The sp^2^ hybridized carbon (C = C) skeleton vibration peak could be seen in GO around 1633 cm^−1^. Compared to GO, rGO shows significant reduction in absorption intensities due to the presence of oxygen containing functional groups like carboxylates, epoxide, and carbonyl compounds, indicating the green reduction of GO to rGO by both *Citrus sinensis* and *Musa acuminata* peel waste extracts. As can be presented in Figures 8(a) and 8(b), the peaks centered at 2854.33 and 2921 76 cm^−1^ in the spectrum of rGO are due to the stretching vibration of H-C-H and -C-H groups of alkanes associated with H-bond as well [44].

FT-IR spectra of TiO_2_ showed the broad band around and below 1000 cm^−1^, which indicates replicate Ti-O-Ti linkage within the TiO_2_ nanopours. Furthermore, the spectra of TiO_2_/rGO exhibited low intensity band frequency compared to the *Citrus sinensis* and *Musa acuminata* stabilized GO and rGO, which is formed by the amalgamation of (Ti-O-Ti) and (Ti-O-C) linkages, owing to the chemical interaction of TiO_2_ with rGO sheets. This analysis confirms the green reduction of GO and coupling with TiO_2_ NPs on the green obtained rGO sheets. In addition to this, the *Citrus sinensis* and *Musa acuminata* template obtained TiO_2_ NPs could be susceptible to the interactions with the functional groups of rGO in the formation of TiO_2/_rGO nanocomposites [47].

### 3.7. Visible Light Photocatalytic Degradation Study of MB

Figures 9(a) and (e) show the changes in the MB absorption spectra during photocatalytic degradation with TiO_2_-2c (a) and TiO_2_-2 m (e) nanophotocatalyst at different solar irradiation times varying from 0 to 60 min. As it can be observed from the figures, the degradation of MB using TiO_2_ only nanophotocatalyst is very low indicating low photocatalytic activity of TiO_2_ only NPs [48]. From the results presented, only 62% and 58.5% of the dye were degraded in the presence of TiO_2_-2c and TiO_2_-2 m nanophotocatalysts, respectively. The low photocatalyst degradation efficiency of TiO_2_only NPs could be attributed to the high electron-hole recombination rate [49].

Figure 9 also depicts photocatalyst degradation of MB of *Citrus sinensis* peel extract mediated synthesized TiO_2_/rGO (b–d) and *Musa acuminata* mediated synthesized TiO_2_/rGO (f–h) nanophotocatalysts using different volume ratios. Among the various TiO_2_/rGO nanocomposite photocatalysts, TiO_2_/rGO-1.5c and TiO_2_/rGO-1.5 m showed the highest degradation efficiency of 94.28% and 94.25%, respectively, after 60 min irradiation.

The results showed that the visible light photocatalytic degradation of MB is dependent on the concentration of rGO composited with TiO_2_ nanophotocatalyst. As supported by the previous report [50], high surface area of the nanocomposite photocatalysts promotes increased dye adsorption on its surface. Furthermore, the improvement in photocatalytic performance of TiO_2_/rGO nanophotocatalysts might also be due to the decrease in the electron-hole recombination rate since rGO in TiO_2_/rGO nanocomposites can act as an electron acceptor.

Reaction kinetics study models for the photocatalytic degradation of MB dye using both TiO_2_ nanocatalysts and TiO_2_/rGO composite nanocatalysts were tested by using first and second order pseudokinetic models. As it can be observed from Figure 10(a), the photocatalytic degradation of MB fit pseudo-first order model with the correlation constant of *R*^2^ = 0.95 min^−1^ for the TiO_2_-2c and *R*^2^ = 0.953 for the TiO_2_-m nanophotocatalysts.

Table 1 represents the corresponding calculated parameters for first order and second order kinetic data model of MB dye degraded by green formed TiO_2_ nanocatalyst and TiO_2_/rGO nanocomposites under visible light irradiation.

Furthermore, the photocatalytic degradation of MB in the presence of green template TiO_2_/rGO green nanocatalysts was found to be fit with pseudo-second order kinetics with rate constant of 0.974 min^−1^ for TiO_2_/rGO-1.5 m [51].

Figures 11(a)–11(c) showed the influence of pH of the solution on the degradation efficiency of methylene blue using TiO_2_/rGO nanophotocatalysts at pH 1, 7, and 13 (strong acid, neutral, and strong base media), respectively. The change in the pH of the solution influences the surface of the nanocomposite catalyst, thereby causing a change in adsorption and the reaction rate [52]. The point of zero charges of the TiO_2_/rGO-1.5c was estimated to be at pH 7 and as a result the photocatalyst surface could possess negative charge at pH > 7 and positive charge at pH < 7. It was observed that when the pH of solution changed from pH 1 to pH 7, the degradation efficiency of the NC increased from 18.1 to 90.7, respectively. The low degradation efficiency of MB in the presence of TiO_2_/rGO nanophotocatalysts at pH 1 could be due to the electrostatic repulsion between the positively charged green nanophotocatalysts surface and the cationic methylene blue, while no such repulsion occurs at pH 7 [10].

The photocatalytic degradation of MB dye in the presence of green template synthesized TiO_2_/rGO nanophotocatalysts was found to be dependent on the pH value. This pH dependence of photocatalyst activity of the NC might be due to its effect on the NC's surface charge, size, and valance and conductance bond positions [53]. As could be depicted in Figure 11(c), the highest degradation of MB dye was obtained at pH 13 with degradation efficiency of 99.4%. This indicates that alkaline pH favored the adsorption of the dye due to the electrostatic attraction between the negatively charged catalyst surface and cationic methylene blue dye. Furthermore, the neutral pH is known as the zero point of charge where the surface of CS mediated synthesized TiO_2_/rGO NCs has no dye concentration [53].

Figure 12 shows the effect of initial MB dye concentration in the presence of *Citrus sinensis* fruit peel extract template synthesized TiO_2_/rGO-1.5c NCs photocatalyst. The effect of initial MB dye concentrations on the photocatalytic efficiency of the TiO_2_/rGO-1.5c was investigated by varying the concentration of MB dye (10, 20, and 30 ppm) while fixing the amount of the photocatalyst NC (30 mg/L) at pH of 7. It has been found that a significant decrease in the percentage of degradation was observed with an increase in the initial dye concentration of MB dye [54]. This might be caused by the saturation of the surface of the green TiO_2_/rGO nanocomposite catalysts. In addition, the decrease in photodegradation with increase in initial concentration of MB might also be caused by the interference for visible light to penetrate and reach the catalyst surface, thereby lowering the production of OH^−^ radicals [55, 56]. Furthermore, the reaction rates were found to be decreased with an increase in concentration of MB with rate constants of 0.04 min^−1^ for 10 mg/L, 0.03 min^−1^ for 20 mg/L, and 0.02 min^−1^ for 30 mg/L (Figure 12(d)).

In order to gain further information on the degradation removal of MB dye, the dosage of green template TiO_2_/rGO-1.5c nanocomposite photocatalyst was also altered in the range of 20 mg/L, 30, and 50 mg/L while keeping the pH and the dye concentration being 7 and 10 mg/L, respectively. As it is depicted from Figures 13(a)–13(c), maximum degradation efficiency of 90.92% and 90.70% was obtained with 50 and 30 mg TiO_2_/rGO-1.5c dosage, respectively, due to increase in the total number of active sites as the dosage of the photocatalyst is increased [57].

The effect of visible light illumination contact time from 0 to 60 min interval was carried out using 20 mg/L aqueous solution of MB dye at pH 7 in the presence of 30 mg TiO_2_/rGO-1.5c.  Figure 14 depicts the effect of contact time on the degradation of MB dye using the optimized pH. The reaction was started in dark condition for 10 minutes to attain sorption-desorption equilibrium between the catalytic surface and the dye.

The result showed a noticeable gradual increase of photocatalytic rate with increasing illumination time. After 60 min, the rate reached its optimum removal efficiency, 94.4%, and a linear relationship between degradation of MB dye and increase in contact time was observed. This is because prolonging irradiation time allows light to fall on the catalyst surfaces and induce formation of photon excited species and enhances the photocatalytic activities [58].

## 4. Conclusions

In the present findings, TiO_2_ NPs and TiO_2_/rGO NCs were effectively synthesized in the presence of peel waste extract of *Musa acuminata* and *Citrus sinensis* as both a green reducing and stabilizing agent. The synthesized NPs and NCs were characterized using TGA/DTA, XRD, SEM, TEM, HRTEM, SAED, UV-DRS, and FTIR analysis. The thermal stability study proved that the synthesized NPs were found to be stable above 550°C. The XRD analysis shows that the average crystalline size of TiO_2_ NPs was calculated as 27.3, 12.1, and 7.3 nm for the TiO_2_-0.5c, TiO_2_-1c, and TiO_2_-2c and 22.4, 16.3, and 13.4 nm for the volume ratios of TiO_2_-0.5 m, TiO_2_-1 m, and TiO_2_-2 m, respectively. The average crystalline size for the various TiO_2_/rGO NCs was found to be 8.4, 15.3, and 7.5 nm and 12.5, 11.4, and 11.2 nm for the TiO_2_/rGO-0.5c, TiO_2_/rGO-1c, TiO_2_/rGO-1.5c, and TiO_2_/rGO-0.5 m, TiO_2_/rGO-1 m, and TiO_2_/rGO-1.5m, respectively. The UV-DRS analysis showed that the energy band gaps were found in the range of 3.17–3.29 and 3.10–3.38 eV for the *Citrus sinensis* and *Musa acuminata* peel waste extract mediated synthesized TiO_2_ NPs, respectively. The energy band gaps of the various TiO_2_/rGO NCs were found in the range of 2.85–3.11 eV and 3.07–3.11 eV for the *Citrus sinensis* and *Musa acuminata* peel waste extract template synthesized TiO_2_/rGO NCs, respectively. Furthermore, FTIR analysis proved the presence of various bioactive molecules in the peel waste extract of the *Citrus sinensis* and *Musa acuminata* such as phenols, flavonoids, carboxylic acids, alcohols, and saturated and unsaturated hydrocarbons. *Citrus sinensis* template obtained TiO_2_ nanocatalyst showed degradation efficiency of 62%, while *Musa acuminate* obtained TiO_2_ nanocatalyst shows a degradation efficiency of 58.2%. Of the various *Citrus sinensis* and *Musa acuminata* peel waste extract based synthesized TiO_2_/rGO nanocomposites, TiO_2_/rGO-1.5c and TiO_2_/rGO-1.5 m showed degradation efficiency of 94.28% and 94.25%, respectively, making the NCs material of interest for environmental remediation applications.

## Figures and Tables

**Figure 1:** Schematic green synthesis procedure of TiO_2_ (1 : 1) NPs in the presence of *Citrus sinensis* peel extract.

**Figure 2:** Diagrammatic synthesis procedure of rGO using *Citrus sinensis* peel extract.

**Figure 3:** TGA/DTA curve of (a) *Citrus sinensis* and (b) *Musa acuminate* mediated synthesis of TiO_2_ NPs.

**Figure 4:** XRD spectra of (a) *Citrus sinensis*-TiO_2_ NPs, (b) *Musa acuminata*-TiO_2_ NPs, (c) *Citrus sinensis*-TiO_2_/rGO NCs, (d) *Musa acuminata*-TiO_2_/rGO NCs, (e) TiO_2_ NPs, rGO c, and TiO_2_/rGO-*Citrus sinensis* NCs, and (f) TiO_2_ NPs, rGO-m, and TiO_2_/rGO-*Musa acuminata* NCs.

**Figure 5:** SEM micrograph of green synthesized rGO/*Citrus sinensis* peel (a), rGO/*Musa acuminata* peel (b), TiO_2_-0.5c (c), TiO_2_-1c (d), TiO_2_-1.5c (e), TiO_2_-0.5 m (f), TiO_2_-1 m (g), TiO_2_-1.5 m (h), TiO_2_/rGO-0.5 (i), TiO_2_/rGO-1c (j), TiO_2_/rGO-1.5c (k), TiO_2_/rGO-0.5 m (l), TiO_2_/rGO-1 m, (m), and TiO_2_/rGO-1.5 m (n).

**Figure 6:** TEM image of TiO_2_/*Citrus sinensis* peel NPs (a), TiO_2_/rGO/*Citrus sinensis* peel NCs (b), TiO_2_*Musa acuminata* peel NPs (c), and TiO_2_/rGO/*Musa acuminata* peel NCs (d). HRTEM image of TiO_2_/*Musa acuminata* (e), TiO_2_/*Citrus sinensis* (f), TiO_2_/rGO/*Musa acuminata* NCs (g), and TiO_2_/rGO/*Citrus sinensis* NCs (h). SAED pattern of TiO_2_/*Citrus sinensis* (i), TiO_2_/Musa acuminata (j), TiO_2_/rGO/*Musa acuminata* NCs (k), and TiO_2_/rGO/*Citrus sinensis* NCs (l).

**Figure 7:** Tauc plot of TiO_2_ NPs and TiO_2_/rGO NCs obtained using CS and MA peel waste extract.

**Figure 8:** FTIR spectra of (a) *Citrus sinensis*, *Citrus sinensis* template synthesized GO, rGO, TiO_2_, and TiO_2_/rGO, and (b) *Musa acuminata*, *Musa acuminate* template synthesized GO, rGO, TiO_2_, and TiO_2_/rGO.

**Figure 9:** Visible light photocatalytic degradation of *Citrus sinensis* and *Musa acuminata* template synthesized TiO_2_ NPs and TiO_2_/rGO NCs.

**Figure 10:** Pseudo-first (a) and pseudo-second (b) order kinetic models for photocatalytic degradation of MB dye using *Citrus sinensis* and *Musa acuminate* template synthesized TiO_2_ NPs and TiO_2_/rGO NCs.

**Figure 11:** Effect of pH (a–c) and % of degradation (d) on the photocatalytic degradation of MB in the presence of TiO_2_/rGO-1.5c NC.

**Figure 12:** Effect of initial concentration of MB in the presence of synthesized TiO_2_/rGO-1.5c NCs green catalyst.

**Figure 13:** Effect of *Citrus sinensis* peel extract mediated synthesized TiO_2_/rGO-1.5c NCs green catalyst dosage on the photocatalytic degradation of MB.

**Figure 14:** Effect of contact time (a) and % of degradation (b) on the degradation of MB using optimized CS peel extracts template TiO_2_/rGO-1.5c NCs green catalyst.

**Table 1:** Calculated parameters for first and second order kinetic data model.

First order (ln(*A*_*t*_/*A*_*i*_) = −*k*_*t*_) data				Second order (1/*A*_*t*_ = *k*_*t*_ + 1/*A*_*o*_) data			
Nanomaterials	Intercept	Slope	*R* ^2^	Nanomaterials	Intercept	Slope	*R* ^2^
Control	−0.098	−0.006	0.955	Control	0.42581	0.00287	0.9802
TiO_2_-2c	−0.01	−0.014	0.95	TiO2-2c	0.37816	0.00846	0.88616
TiO_2_/rGO-0.5c	−0.051	−0.024	0.83	TiO2/rGO-0.5c	1.09519	0.07185	0.85933
TiO_2_/rGO-1c	−0.94	−0.03	0.8	TiO2/rGO-1c	1.04936	0.06333	0.85933
TiO_2_/rGO-1.5c	−1.07	−0.036	0.828	TiO2/rGO-1.5c	1.09519	0.07185	0.85933
TiO_2_-2 m	−0.098	−0.011	0.953	TiO2-2 m	0.41428	0.00688	0.8976
TiO_2_/rGO-0.5 m	−0.084	−0.02	0.66	TiO2/rGO-0.5 m	0.5731	0.03761	0.81955
TiO_2_/rGO-1 m	−0.75	−0.02	0.79	TiO2/rGO-1 m	0.8615	0.03209	0.92895
TiO2/rGO-1.5 m	−1.07	−0.035	0.819	TiO_2_/rGO-1.5 m	1.31106	0.09163	0.97396

## Data Availability

The necessary data such as TGA/DTA, XRD, UV-DRS, UV-visible absorption spectra, FTIR spectra, SEM, TEM images, HRTEM images, SAED patters, and the photocatalytic degradation study used to support the findings of this study are included in the article.
